# Medical Image Diagnostic Value of Computed Tomography for Bladder Tumors

**DOI:** 10.1155/2021/3781028

**Published:** 2021-11-16

**Authors:** Lin Li, Risu Na, Tao Mi, Hao Cheng, Lili Ma, Guojun Chen

**Affiliations:** ^1^Graduate School of the Affiliated Hospital of Qinghai University, Graduate School, Xining, Qinghai 810000, China; ^2^Qinghai University, Xining, Qinghai 810000, China; ^3^Department of Urology, Affiliated Hospital of Qinghai University, Xining, Qinghai 810000, China

## Abstract

**Objective:**

To study computed tomography (CT) imaging characteristics of bladder tumors, to explore the value of CT in tumor diagnosis, and to identify the relevant factors of CT missed diagnosis so that medical staff can be more accurate in the diagnosis of bladder tumors.

**Methods:**

To retrospectively analyze the CT manifestations of 153 bladder tumor cases confirmed by paraffin pathology in our hospital and to study the difference between the benign and CT imaging features. CT indicators mainly include the number, location, morphology, calcification, bladder wall smoothness, CT value, degree of enhancement, and invasion of surrounding tissues and organs. Then, we retrospectively analyze 17 cases of CT missed diagnosis of bladder tumors, analyze related factors, and discuss the role of CT in the diagnosis of bladder tumors.

**Results:**

This study has shown that with the help of CT images, the diagnosis rate of bladder tumors has been greatly improved. Of the 153 patients studied, noninvasive urothelial carcinoma accounted for 18.95% of all benign and malignant bladder tumors, invasive urothelial carcinoma accounted for 67.93%, prostatic metastatic carcinoma and inflammatory myofibroblastoma accounted for 8.47%, pheochromocytoma accounted for 1.31%, inverted papilloma accounted for 1.31%, tubular choriocarcinoma accounted for 0.63%, and endocystitis accounted for 1.31%. In addition, the blood supply level, CT index bladder wall smoothness, and CT value are also statistically significant (*P* < 0.05).

**Conclusions:**

CT is of high value in the diagnosis of bladder tumors, and benign and malignant bladder tumors have CT and CT imaging features. The size of bladder tumors is related to the missed diagnosis rate of CT. The application of CT examination technology can improve the accuracy of diagnosis of bladder tumors.

## 1. Introduction

The bladder tumor is the most common tumor in the genitourinary system, generally more men than women [1, 2]. Bladder tumors mostly come from epithelial tissues, mainly including transitional epithelial cancer, adenocarcinoma, squamous cell carcinoma, and inverted papilloma. Nonepithelial bladder tumors mainly include inflammatory myofibroblastoma, pheochromocytoma sarcoma, hemangioma, and lymphoma. Bladder cancer is the most common bladder cancer [3–5].

Bladder tumors are the most common tumors in the urinary system, and bladder cancers are the most common lesions of bladder tumors. At present, the incidence of bladder cancer ranks 9th among common tumors worldwide, and the mortality rate ranks 13th. It accounts for about 4% of all malignant tumors in the whole body and is the 5th cause of death in men over 75 years old. The most common sites are the bladder triangle, the lateral wall, and the posterior wall, with multicentric lesions being the most common morphology. Academically, the lesions are mostly local cauliflower-like protrusions [6–9]. Therefore, early detection and early diagnosis are crucial to the treatment and prognosis of the disease.

The main causes of bladder cancer are as follows. (1) Studies have shown that long-term exposure to aromatic chemicals can cause an increase in the incidence of bladder cancer, so those chemical factory workers are a high-risk group for bladder cancer. (2) Long-term smokers are also a high-incidence group of bladder tumors, but the specific pathogenic mechanism needs further study. (3) The bladder mucosa has been subjected to local long-term irritation, such as chronic infection and bladder stones. (4) Certain drugs and parasitic diseases have a high correlation with the occurrence of bladder cancer and have already attracted clinical attention. The most common clinical symptom of bladder cancer is painless gross hematuria throughout the process, and sometimes, it can also be manifested as microscopic hematuria. Diagnosing bladder cancer based on clinical symptoms alone has a large error because the hematuria is often not directly proportional to the tumor. Therefore, an auxiliary examination is needed to clarify the condition of the tumor. CT is a commonly used examination method [10, 11].

In the clinical diagnosis and treatment of bladder diseases, electronic computed tomography (CT) examination is an effective localization examination method. Compared with ultrasound, CT examination can better show the tissue structure around the bladder, whether there is an invasion of the surrounding tissue, the extent of invasion, and pelvic or retroperitoneal lymph node metastasis. Enhanced CT imaging can better reflect the blood supply of the lesion, and through the reconstruction of the target blood vessel image, the blood vessel structure is clearly displayed, which is of great significance to the diagnosis and treatment of the lesion. Past studies have shown that 64-slice CT examination has a sensitivity of about 85% and a specificity of about 85% for the diagnosis of bladder cancer. Thin-layer enhanced CT scanning can be used for preoperative diagnosis and staging of bladder cancer, which is of great value for the rational choice of clinical treatment and prognostic evaluation.

Nowadays, CT urography has developed rapidly and has been widely used in the clinical work of bladder tumor diagnosis and treatment. CT is a method of observing CT scan images before and after intravenous injection of the contrast agent. It is a fast, simple, noninvasive, and comprehensive urinary tract examination method. It can detect bladder lesions and describe their relationship with adjacent tissues and organs. The relationship between the discovery of lymph node metastasis outside the bladder and the distant metastasis of the tumor has now become an essential test in the diagnosis and treatment of bladder cancer.

With the development of CT instruments, the combination of some new technologies can improve the diagnosis rate of bladder tumors. Studies have shown that the low-emission CT virtual cystoscope has a sensitivity of 100% for bladder tumors larger than 0.5 cm, the bladder tumors at 0.5 cm can also achieve high sensitivity, and the average radiation absorption equivalent (6.9 mSv) is significantly less than that of conventional 16-row spiral CT. Spiral CT and its reconstruction technology can show the enhancement of the mass and the thickening of the bladder wall, which is of great value in the diagnosis of bladder cancer [12]. Studies have shown that multislice spiral enhanced CT dual-phase scanning combined with virtual endoscopic imaging is of great value for preoperative clinical staging of bladder cancer. The staging accuracy rate is 94.5%. When the tumor is limited to the bladder wall (≤T2b), the diagnosis accuracy rate is 91.2%; when the tumor invades the outer structure of the bladder wall (≥T3), the diagnosis accuracy rate is 100%. In recent years, cone-beam CT has been used to guide radiation therapy for bladder cancer, and it has opened up new fields for the application of imaging to bladder cancer.

Nowadays, CT examination has been more and more widely used in the clinic. As a commonly used imaging examination method, CT can not only observe the location, density, size, shape, and boundary of the lesion, the CT value, and the degree of enhancement when detecting bladder space-occupying lesions but also understand whether the lesion is cystic or bleeding, calcified, etc. At the same time, it can better show the structure of the surrounding bladder, whether there is an invasion of the surrounding tissue, the extent of invasion, and pelvic or retroperitoneal lymph node metastasis. It can also understand whether there are enlarged lymph nodes and abnormal changes around the bladder. By rebuilding the target blood vessel image, we can then display the vascular structure in the diagnosis of bladder cancer, tumor staging, and selection of treatment methods [13, 14].

## 2. Materials and Methods

### 2.1. Research Subjects

We select patients who underwent urinary bladder enhancement CT examination in our hospital from January 2016 to July 2020 before undergoing surgical treatment in the urology department of our hospital, and we exclude cases with no clear pathological results. Finally, 153 patients were included, including 127 males and 26 females, with a male to female ratio of 4.88 : 1. The age range is 19-92 years, with an average age of 62.44 ± 11.19 years and a median age of 63 years. All tumors were confirmed by paraffin pathology.

### 2.2. Research Methods

#### 2.2.1. Equipment Selection

*CT instrument:* 16-layer and 64-layer LightSpeed CT scanners of GE company are used.

*Contrast agent:*the agent used is itopride (35% or 37%), the dose is 100 ml, the injection rate is 2-3 ml/s, and it is injected through the peripheral vein [15].

#### 2.2.2. CT Inspection Method

The patient fasted for 3 to 5 hours before examination, the bladder was moderately filled, the supine position was taken, the scan range was from the diaphragm top to the pubic symphysis, and the breath was scanned after breathing in deeply. Scanning parameters are as follows: layer thickness 2.5~5.0 mm and layer distance 1.25~5.0 mm; CT scan was first, and then we injected iodine via the superficial elbow vein (iodine 350 mg/100 ml or iodine 370 mg/100 ml, 35% or 37%). The dose is 100 ml, and the injection rate is 2 to 3 ml/s. We took the enhanced early scan 20-40 s after injection and the enhanced late scan 40-60 s. All images are stored in this machine or uploaded to an image archiving and communication system for retrospective analysis.

In this study, we observed the number, location, shape, presence or absence of calcification, bladder wall smoothness at the junction of the lesion, and tumor invasion of surrounding tissues and organs on CT images and recorded the CT value and degree of enhancement of the lesion.

The specific inspection categories are as follows:

*(1) Number.* According to the number of lesions, it is divided into single and multiple.

*(2) Location.* According to the growth position of the lesion in the bladder, it is divided into the anterior wall, posterior wall, and top, bottom, and side walls.

*(3) Morphology.* According to the shape of the lesion, it is divided into the bulge type and infiltration type.

*(4) CT Value.*We determine the maximum level of the lesion, measured with a 5 mm^2^ circular area, using the Hounsfield unit (Hu).

*(5) Bladder Wall Smoothness.* According to the smoothness of the bladder wall at the junction of the lesion and the bladder, it is divided into smooth and nonsmooth.

*(6) Judgment Method of Calcification.* If the CT value of the plain scan exceeds 100 Hu, it is regarded as calcification.

*(7) Degree of Enhancement.* According to the results of the lesion enhancement scan compared with the surrounding normal bladder wall, it is divided into two categories: no significant enhancement and significant enhancement.

*(8) Infiltration and Metastasis of Surrounding Tissues.* According to the relationship between the bladder tumor and ureter and other adjacent tissues and lymph node metastasis, it is divided into no infiltration metastasis and infiltration metastasis.

#### 2.2.3. Analysis Content

Two professionally trained doctors performed retrospective analysis of the images without knowing the pathological results. If there is any inconsistency between the qualitative data, the two will negotiate and record the data after reaching an agreement. According to the pathological results of paraffin, the cases of CT missed diagnosis were analyzed. In CT detection, the size, number, morphology, echo level, calcification, bladder wall continuity, and invasion of surrounding tissues and organs of the lesion were observed. We observed the size, number, morphology, presence or absence of calcification, bladder wall smoothness at the junction of the lesion, and tumor invasion of surrounding tissues and organs on CT images and recorded the CT value and degree of enhancement of the lesion.

### 2.3. Statistical Methods

The data in this study are statistically processed by software SPSS 20.0. Normal measurement data is expressed by (*x* ± *s*), the comparison of count data between groups is the *X*^2^ test, and the count data is expressed by the number of cases (*n* (%)). The *t*-test was used for comparison between the two groups, with *P* < 0.05 indicating that the difference was statistically significant.

## 3. Results

### 3.1. Pathological Results and General Conditions

For the study of 153 patients, according to the paraffin pathological diagnosis, the pathological types were divided into the following: (1) 145 cases of malignant bladder tumors: 29 cases of noninvasive urothelial carcinoma, including 2 cases of carcinoma *in situ*, and noninvasive urothelial carcinoma with 1 case of focal squamous cell metaplasia and one case of noninvasive urothelial carcinoma with glandular differentiation, 104 cases of invasive urothelial carcinoma, including 1 case of invasive urothelial carcinoma with adenocarcinoma differentiation, and 12 cases of prostatic metastatic carcinoma; and (2) 8 cases of benign bladder lesions: 2 cases of pheochromocytoma, 2 cases of inverted papilloma, 1 case of tubular choriocarcinoma, 1 case of inflammatory myofibroblastoma, and 2 cases of endocystitis. The pathological results of 153 patients are summarized in Table 1.

Among the 153 patients studied, there were 8 benign bladder tumors, with an average age of 52.30 ± 14.56 years, and 145 malignant bladder tumors, with an average age of 66.14 ± 12.10 years. The difference was statistically significant (*P* < 0.01), and the summary is shown in Table 2. The study found that the average age of patients with malignant bladder tumors is significantly greater than the average age of patients with benign bladder tumors. The gender distribution of benign and malignant tumors was not statistically significant.

### 3.2. CT Imaging Analysis

In order to more intuitively demonstrate the role of CT examination in the diagnosis of bladder tumors, this study selected CT examination images of multiple patients for analysis. The schematic diagram of CT examination of multiple patients and their corresponding pathological conditions are shown below. Through the four images in Figure 1, we can draw the CT image to determine the growth position of the bladder tumor and visually observe the performance of the tumor lesion.

### 3.3. CT Diagnosis of Benign and Malignant Bladder Tumors

In this group of studies, there were 5 benign single lesions, 3 multiple lesions, 100 malignant single lesions, and 45 multiple lesions. There was no statistical difference between the two (*X*^2^ = 0.21, *P* > 0.05). There is no obvious correlation between the benign and malignant tumors and their number (see Table 3).

According to the CT detection results, the location of the tumor was located. The results showed that the posterior walls of the bladder were the highest site of tumors, followed by the side of the bladder. See Table 4 for the distribution of the growth sites of good and bad lesions. Benign bladder tumors were located in the following: 1 at the anterior wall of the bladder, 3 at the posterior walls, 2 at the top, 1 at the bottom, and 1 at the lateral walls. Malignant bladder tumors were located in the following: 15 at the anterior walls, 75 at the posterior walls, 3 at the top, 2 at the bottom, and 50 at the lateral walls. The growth position of benign and malignant tumors is statistically different (*P* < 0.05). Malignant tumors occur most frequently on the posterior wall of the bladder, while benign tumors are relatively rare on the side wall of the bladder. The distribution of the growth positions of benign and malignant tumors is shown in Table 4, and the statistical diagram of tumor growth positions is shown in Figure 2.

The results showed that the average CT scan value of malignant tumors was 36.26 ± 7.97 Hu, range 17~58 Hu, and the average enhancement (arterial phase) CT value was 70.47 ± 17.57 Hu, range 29~131 Hu; for the average scan of benign tumors, the CT value was 41.11 ± 12.68 Hu, ranging from 24 to 77 Hu, and the average enhancement (arterial phase) CT value was 62.26 ± 27.36 Hu, ranging from 31 to 121 Hu. The average CT scan of benign and malignant tumors and the enhancement (arterial phase) CT value difference were statistically significant (*P* = 0.02 and *P* = 0.01). We analyzed the morphology of the lesion and the smoothness, calcification, and enhancement of the bladder wall at the junction of the lesion. After the statistical results, it was found that the smoothness of the connection between the tumor and the bladder wall and the degree of tumor enhancement between the benign and malignant groups were statistically significant (*P* < 0.05). It shows that the benign and malignant tumors are related to the above CT features. Malignant tumors are more likely to be roughened bladder walls. The enhanced CT showed that most of the malignant tumors were significantly strengthened, and the difference in the degree of enhancement of benign and malignant tumors was statistically significant. There was no statistically significant difference between the benign and malignant groups in the morphology of the tumor and the presence or absence of calcification (*P* > 0.05).

## 4. Discussion

CT examination can allow us to analyze the degree of enhancement of the lesion, understand whether the lesion is cystic or calcified, and make a certain diagnosis for bladder-occupying diseases. Moreover, CT has an important reference value for the selection of disease treatment methods by observing the surrounding tissue, pelvic or abdominal lymph node metastasis, and metastasis status [16].

CT is the use of an X-ray beam to scan a certain thickness of a certain part of the human body and then input it into the computer for processing to form a CT image. CT examination can observe the CT value and degree of enhancement of the lesion, understand whether the lesion is cystic or calcified, and make a certain diagnosis for bladder-occupying diseases. Moreover, CT has a high value for the diagnosis of bladder tumors by observing the surrounding tissue, pelvic or abdominal lymph node metastasis, and metastasis status [17–20].

However, CT examination also has certain deficiencies, and it is not easy to distinguish the lesions that do not cause bladder wall thickening, which may cause missed diagnosis. The accuracy of CT examination has a certain correlation with the size of bladder tumor lesions, and the detection accuracy decreases for tumor diameters less than 10 mm [12, 21, 22]. The results of this study show that CT has a missed diagnosis rate of 64.71% for bladder tumors smaller than 10 mm, which is consistent with previous literature reports [23–28]. However, the combination of some professional new technologies in clinical work now can improve the diagnosis rate of CT for microbladder tumors. Studies have shown that the low-radiation CT virtual cystoscope has a sensitivity of 100% for bladder tumors larger than 5 mm and can also achieve higher sensitivity for bladder tumors smaller than 5 mm. On the other hand, CT is most likely to miss a tumor in the top of the bladder, followed by the side wall and bottom. For tumors in the anterior wall of the bladder, the CT diagnosis rate in this study was 100% [29–31].

All cases in this study were confirmed by paraffin pathology, and the male to female ratio was 4.88 : 1, which was similar to previous reports in the literature [32, 33]. In the identification of benign and malignant bladder tumors, this study first found that the average age of patients with benign and malignant bladder tumors was statistically different. The average age of patients with malignant bladder tumors was higher than that of patients with benign bladder tumors. In addition, in this group of cases, the posterior wall of the bladder is the most frequent site of tumors, followed by the anterior and side walls of the bladder, and the bottom wall and top of the bladder have fewer tumors. The growth position of benign and malignant tumors does not also have a statistical difference (*P* < 0.05). Malignant tumors and benign tumors occur most on the posterior wall of the bladder, and both of them are relatively rare on the bottom wall of the bladder.

## 5. Conclusion

In summary, CT has a certain value in the differentiation of benign and malignant tumors of the bladder, but the specific imaging indicators are relatively few. The bladder tumors of different pathological types have certain self-imaging characteristics in CT imaging. So CT examination can further improve the accuracy of preoperative diagnosis of bladder tumors.

The missed diagnosis of CT examination has a certain correlation with the size of bladder tumor lesions and the gender difference, and there was no significant correlation between age, tumor number, and growth location. CT examination can play a certain role and improve the diagnosis of bladder tumors.

## Figures and Tables

**Figure 1:** CT medical image of the patient depicting the following: multiple lesions in the bladder (a); round bulge-like lesions in the bladder (b); bladder wall unevenness at the junction of the lesions (c); plaque calcification in the lesions (d).

**Figure 2:** Statistics of the tumor growth number and position (the *X* axis is the growth position of the bladder tumor, and the *Y* axis is the growth number of the bladder tumor).

**Table 1:** Pathological diagnosis results.

Pathological type	Number of cases	Percentage (%)
Noninvasive urothelial carcinoma	29	18.95
Invasive urothelial carcinoma	104	67.93
Prostatic metastatic carcinoma	12	7.84
Pheochromocytoma	2	1.31
Inverted papilloma	2	1.31
Tubular choriocarcinoma	1	0.63
Inflammatory myofibroblastoma	1	0.63
Endocystitis	2	1.31
Total	153	100

**Table 2:** Average age and sex distribution of patients with benign and malignant bladder lesions.

		Benign tumor (*n* = 30)	Malignant tumor (*n* = 132)	*P* value
Gender	Male	5	122	0.60
	Female	3	23	
Age		52.30 ± 14.56	66.14 ± 12.10	≤0.01

**Table 3:** Single multiple cases of benign and malignant lesions.

		Benign	Malignant	Total	*X* ^2^	*P* value
Number	Single	5	100	105	0.21	0.65
	Multiple	3	45	48		

**Table 4:** Distribution of benign and malignant bladder tumor growth locations.

		Benign	Malignant	Total	*X* ^2^	*P* value
Position	Anterior wall	1	15	16	16.28	0.03
	Posterior wall	3	75	78		
	Top	2	3	5		
	Bottom	1	2	3		
	Side wall	1	50	51		

## Data Availability

The image data used to support the findings of this study have been deposited in the International Cancer Genome Consortium (ICGC) (https://dcc.icgc.org/).
